The article "Physicians' Attitude towards Electronic Medical Record Systems: An Input for Future Implementers" was published in 2021. Journal: Biomed Res Int.

# Physicians' Attitude towards Electronic Medical Record Systems: An Input for Future Implementers

**DOI:** 10.1155/2021/5523787

**Published:** 2021-08-28

**Authors:** Mulugeta Hayelom Kalayou, Berhanu Fikadie Endehabtu, Habtamu Alganeh Guadie, Zeleke Abebaw, Kassahun Dessie, Shekur Mohammed Awol, Nebyu Demeke Mengestie, Abraham Yeneneh, Binyam Tilahun

**Affiliations:** Department of Health Informatics, Institute of Public Health, University of Gondar, Ethiopia

## Abstract

**Background:**

Electronic medical record (EMR) systems offer the potential to improve health care quality by allowing physicians real-time access to patient healthcare information. The endorsement and usage of EMRs by physicians have a significant influence on other user groups in the healthcare system. As a result, the purpose of this study was to examine physicians' attitudes regarding EMRs and identify the elements that may influence their attitudes.

**Method:**

An institutional-based cross-sectional study design supplemented with a qualitative study was conducted from March 1 to April 30, 2018, among a total of 403 physicians. A self-administered questionnaire was used to collect quantitative data. The validity of the prediction bounds for the dependent variable and the validity of the confidence intervals and *P* values for the parameters were measured with a value of less than 0.05 and 95 percent of confidence interval. For the supplementary qualitative study, data were collected using semistructured in-depth interviews from 11 key informants, and the data were analyzed using thematic analysis.

**Result:**

Physicians' computer literacy (CI: 0.264, 0.713; *P*: 0001) and computer access at work (CI: 0.141, 0.533, *P*: 0.001) were shown to be favorable predictors of their attitude towards EMR system adoption. Another conclusion from this study was the inverse relationship between physicians' prior EMR experience and their attitude about the system (CI: -0.517, -0.121; *P*: 0.002).

**Conclusion:**

According to the findings of this study, physicians' attitudes regarding EMR were found moderate in the studied region. There was a favorable relationship between computer ownership, computer literacy, lack of EMR experience, participation in EMR training, and attitude towards EMR. Improving the aforementioned elements is critical to improving physicians' attitudes regarding EMR.

## 1. Introduction

Different information communication technologies (ICTs) are being implemented and used in health care for facilitating the service and strengthen the health system. Among them, the electronic medical record (EMR) system is one of the common systems which helps to store, analyze, and access health-related information of patients [1]. Based on different studies in different settings, the EMR system is perceived as the way to advance information exchange, saving time, data confidentiality, and decision makings [2, 3]. Because of those potential benefits, electronic medical record systems are rapidly being implemented in healthcare settings of many countries, including in the low-resource setting countries [4–7].

The article "Physicians' Attitude towards Electronic Medical Record Systems: An Input for Future Implementers" was published in 2021. Journal: Biomed Res Int.

Currently, the Ethiopian Federal Ministry of Health (EFMOH) has considered developing and formulating a national eHealth strategy that realize standardization and implementations of national eHealth systems like health data warehouse, Health Net, tele education, telemedicine, human resource information system, electronic health information management system, woreda-based planning system, and health integrated financial information systems including EMR systems [8, 9]. The Ministry had been implemented an EMR system called SmartCare, introduced with support of Tulane University Technical Assistance Project in Ethiopia (TUTAPE). The system had deployed in different wards like laboratory, registration room, OPD, pharmacy, antiretroviral therapy (ART), and maternal and child health units [10, 11].

Even though the implementation and success rate of EMR is good in developed and highly resourced countries [2, 12, 13], the dissemination and the success rate of EMR in resource-limited countries are still in the embryonic stage [12, 14, 15]. Like other developing nations, though there are high expectations and interests in EMRs in Ethiopia, their overall implementation rates are relatively low and fronting several problems [5]. For instance, they are seen as contrary to a physician's traditional working style, and they require a greater competence in dealing with different computer-related skills like typing [6]. Some physicians were asking for implementers and high-level managers for the assignment of IT personnel who could help them to record paper-based patient histories to the newly introduced SmartCare system since they were expected to document both on paper and within the SmartCare system [10–12, 15].

Besides to the computer-related literacy, exploring end user attitudes and expectations of the fast-developing eHealth services helps to understand the factors that influence adherence to such tools in health care [16]. Good understanding of user's attitude about the system was found the key factor needed to make EMR systems adopt easily. Studies identified that even good technology could be fallen if the intended users have not a positive attitude towards the system [17]. According to some studies [7], the slow rate of EMR implementation suggests that resistance among physicians was strong because Physicians are the main frontline user-group of EMRs. Even though most physicians generally perceive that electronic-based health information systems can help to eliminate the burden of paper-based documentation and the inaccessibility of patient data in life-threatening situations, they also get easily disappointed when an introduced system does not meet their expectations [18–21]. Especially in low-resource countries like Ethiopia, where physician to patient ratio is too high, one to 17,000 people, and a single physician clerked hundreds of patients per day [22, 23], implementing and succeeding in health information systems like EMRs without physicians favorable attitude is unthinkable. Studies showed that the physicians' support and use towards EMRs have a great impact on other user-groups in healthcare system, such as administrative and supportive staff including nurses [24, 25]. Concerning this purpose, several studies have been conducted on the physician's attitude towards electronic-based health information systems like EMRs [26–31]. But when we went through the studies conducted on the physician's attitude to EMRs in Ethiopia, it was deficient and not investigated well. Besides, the findings from the developed world were found incomparable to our setting, which is with low organizational and technical infrastructure.

The article "Physicians' Attitude towards Electronic Medical Record Systems: An Input for Future Implementers" was published in 2021. Journal: Biomed Res Int.

As a result, the purpose of this study was to fill this evidence vacuum by analyzing physicians' attitudes regarding EMRs and the predictive factors that may influence their attitudes. As a result, the findings will have an influence on future adoption success and physician acceptability of EMRs systems in the region.

## 2. Materials and Method

### 2.1. Study Design and Setting

An institutional-based cross-sectional quantitative study supplemented with qualitative approach was conducted from March 1 to April 30, 2018, at the five referral hospitals in Amhara regional state, Ethiopia. The State of Amhara is located in the North Western and North Central part of Ethiopia. The region has five referral hospitals, namely, University of Gondar, Debre Markos, Felege Hiwot, Dessie, and Debre Berhan Referral Hospitals. Each hospital serves a catchment area of more than four million people. The overall existing EMR utilization in the University of Gondar referral hospital was 46.5% [14]. In all the referral hospitals, there is EMR (SmartCare) system implementation history with a plan of expanding it to other primary and general public hospitals in the region. Currently, the system is used only to register patient's sociodemographic and some clinical data at the triage level and to quickly identify and locate patient history cards. Currently, the Ethiopian Ministry of Health is on the way to replace it with a new system called District Health Information System (DHIS2). The new system helps to aggregate regularly collected data across all of the public health facilities of the country [32].

The article "Physicians' Attitude towards Electronic Medical Record Systems: An Input for Future Implementers" was published in 2021. Journal: Biomed Res Int.

### 2.2. Study Population

The study population includes general practitioners, residents, specialists, and subspecialists who are working at Amhara regional state referral hospitals of Ethiopia. Physicians who had less than 6 months of work experience and residents who were not permanent staffs of the selected hospitals were excluded from the study because those physicians could face difficulty to answer organizational-related questions that could possibly affect their attitude to EMRs.

### 2.3. Sample Size and Sampling Procedure

All the 488 physicians who were working in the five referral hospitals (243 at University of Gondar Hospital, 53 at Debre Markos Hospital, 64 at Felege Hiwot Hospital, 80 at Dessie Hospital, and 48 at Debre Berhan Hospital) were included in the study for higher precision and accuracy.

### 2.4. Data Collection Tools and Procedures

Data were collected by trained data collectors using a pretested, structured, and self-administered questionnaire, which was adopted from different literatures [15, 33–35]. The tool was prepared and distributed in English language. Pretest was conducted on a similar setting at Zewditu referral hospital, Addis Ababa Ethiopia before the actual data collection time on 5% of the sample size in order to check the reliability of the instrument, to estimate the time needed to collect data and to modify the questionnaire accordingly. Using the data obtained from the pretest, the questionnaire was checked for internal consistency using the Cronbach alpha test. The reliability for attitude questions had a Cronbach's alpha value of 0.95. These values indicate that the questionnaire has very good reliability. The major contents of the tools were sociodemographic variables, technical, and organizational variables.

To measure the level of attitude towards EMR, fifteen questions were asked. Each attitude question is graded on a five-point scale (strongly agree coded as five, agree coded as four, neutral coded as three, disagree coded as two, and strongly disagree coded as one). Then, using an arithmetic mean, the respondents' scores for the attitude questions were calculated. The linear regression method was used to determine the relationship between the dependent variable and the independent variables. Respondents who can use at least basic Microsoft Office products (MS Word, PowerPoint, and Excel, Access, and Internet services) were also deemed computer literate [15].

The article "Physicians' Attitude towards Electronic Medical Record Systems: An Input for Future Implementers" was published in 2021. Journal: Biomed Res Int.

Six bachelor's degree holder nurses and two general practitioners were recruited as data collectors and supervisors, respectively. Two days of training was given for data collectors and supervisors on the prepared data collection tool, participant rights, data confidentiality, and the general objective of the study. The supervisor's role was coordinating the data collection process and reporting the data collection progress to principal investigator.

For supplementary qualitative data, an in-depth interview was conducted in local language (Amharic) using a semistructured interview questions. Of the 20 physicians who agreed to participate, 11 were interviewed. The 11 key informant in-depth interviews were conducted until the information got saturated. All the elven participants for the in-depth interview part were department heads from different units, who can represent the other study subjects, and they were given strict guarantees of anonymity regarding the data that were collected and we also took written informed consent from all the participants. The interview was conducted by the principal investigator (MHK). The interviews conducted with the participants varied in the length from 25 min to 45 min with the average interview length of 36 min. Probing questions were used to get additional depth when necessary for understanding any of the attitude factors. Besides, all the divergent views raised by the participants were resolved during the interview, with principal investigator (MHK). Audio recorder was used during the interview, which then was transcribed for analysis.

### 2.5. Data Processing and Analysis

Epi-info version 7 was used to enter data from respondents, which was then exported to SPSS version 20 for additional analysis. Although heteroscedasticity does not create bias in the coefficient estimates, it does make them less exact; lesser precision increases the chance that the coefficient estimations are farther from the true population value. The notion of “Robust standard errors” was utilized to remedy standard errors caused by model misspecification. One of the assumptions of linear regression modeling is homoscedasticity. It is necessary to guarantee the accuracy of the estimates, the validity of the prediction bounds for the dependent variable, and the validity of the confidence intervals and *P* values for the parameters. Huber-white tests for heteroscedasticity had a significance value of 0.002. Finally, the variables with significant associations were identified using the significance value for the parameter estimate with a robust standard error of less than 0.05 and a confidence interval of 95%. The general linear method was used to determine the Huber-White standard errors. As a result, generalized linear models and generalized estimating equations provide reliable standard errors. These are the original Huber-White linear model estimators. To conduct the general linear procedure in the SPSS, we followed on analyze > generalized linear models > generalized linear models for a standard model with independent observations. Using open code version 4.3, thematic analysis was performed to analyze the supplemental qualitative section. The interview guide was primarily concerned with organizational and technological issues that may influence physicians' attitudes regarding EMR systems. As a result, themes were created based on the preset categories as outlined in the interview guide.

The article "Physicians' Attitude towards Electronic Medical Record Systems: An Input for Future Implementers" was published in 2021. Journal: Biomed Res Int.

## 3. Result

### 3.1. Sociodemographic Characteristics of the Physicians

Out of 488 Physicians who were approached for the study, 403 of them participated in the study with a response rate of 82.5%. From the total of (*n* = 403) respondents, 212 (52%) of them were academic physicians and the majority of the 338 (83.9%) were males and more than half of the 226 (56.1%) had their own computer. And the mean age of the respondents was 33.9 years with a standard deviation of ±4.89 years (Table 1).

### 3.2. Technology-Related Variables of Physicians

The majority of the study participants 286 (71.0%) were computer literate. About 185 (45.9%) and 245 (60.8%) of the study participants had previous EMR experience and were taking EMR training, respectively. In addition, about 245 (60.8%) of the participants prefer EMR over a paper-based systems (Table 2).

### 3.3. Organizational-Related Variables on Physician's Attitude towards EMR

More than half of respondents 235 (58.3%) believe that the hospital administration involves physicians in EMR activities and about half of the respondents 212 (52.6%) had computer access in their working area (Table 3).

### 3.4. Attitude of Physician's towards Electronic Medical Record Systems

Of the total 403 participant physicians, 235 (58.3%) of them had scored more than and equal to the neutral value. All the attitude questions, the fifteen Likert scale questions, were computed into a single value using an arithmetic mean value.

### 3.5. Factors Associated with Physicians' Attitude towards EMR Systems

After controlling for other variables, the correlation coefficient value of the analysis shows that physicians' computer ownership, computer literacy, lack of prior EMR experience, participation in EMR training, and computer access at work were significantly associated with physicians' attitudes towards electronic medical record systems.

The article "Physicians' Attitude towards Electronic Medical Record Systems: An Input for Future Implementers" was published in 2021. Journal: Biomed Res Int.

In this study, physicians' computer ownership was found a significant factor for having a favorable attitude towards EMR systems with a confidence interval of (CI: 0.037, 0.458) and significance value 0.021. In addition, taking an EMR training (CI: 0.159, 0.559, *P*: 0.0001) was found as a positive predictive factor to the system.

Physicians' computer literacy (CI: 0.264, 0.713; *P*: 0001) and computer access at workplace (CI: 0.141, 0.533, *P*: 0.001) were also found a positive predictive factors for the physicians' attitude towards EMR systems use. The other finding from this study was the opposite association of physicians' previous EMR experience and their attitude towards the system (CI: -0.517, -0.121; *P*: 0.002) (Table 4).

### 3.6. Qualitative Results

There were seven males and four females among those who took part in the interviews. Participants were 35 years old on average. Participants ranged in age from 28 to 50 years old. Physicians who can perform basic computer tasks have a better attitude towards using EMRs, according to all key informants. Physicians with computer access were also more comfortable with computer-based information systems and had a better understanding of the benefits of EMR systems, according to the interviews.

Furthermore, the majority of respondents claimed that the previously introduced EMR system had inadequate system architecture and used unstandardized medical terminology, causing care providers' attitudes of EMR systems to be warped. Another issue raised by participants was that in a work environment with a high patient load and low computer literacy among physicians, the difficulty of typing patient-related history on keyboards reduces physician-patient interaction, which may affect attitudes towards EMR systems. The four most prevalent themes that emerged from the in-depth interviews with key informants and qualitative remarks from the written questionnaires were (1) basic computer literacy, (2) prior EMR experience, (3) taking an EMR training, and (4) computer access at work.

#### 3.6.1. Basic Computer Literacy

Physicians who could perform basic computer tasks were shown to have a positive attitude about EMR. Participants who use computers on a regular basis gained a strong understanding of the system. In a word of 33-year-old male participant:

*“I use a computer to prepare PowerPoint presentations and to acquire new knowledge in my field of expertise. This simplifies my life. It (EMR) would be extremely useful in a variety of ways and save a significant amount of time. It is likely to improve patient care by avoiding problems associated with illegible handwriting and facilitating patient information access...”*

The article "Physicians' Attitude towards Electronic Medical Record Systems: An Input for Future Implementers" was published in 2021. Journal: Biomed Res Int.

#### 3.6.2. Previous EMR Experience

Electronic medical record systems may contradict views about how health care should be structured; employing physicians to input data may be inefficient and viewed as degrading; and clinicians and management may need to learn how to use certain software, which may be frustrating. These challenges are exacerbated if the system is not in sync with the organization's work culture. One female physician, identified as “31,” described her past encounter with EMR as follows:

*“I used to use an EMR system that used broad terms rather than specific disease terminologies. This system made our job difficult because it did not support disease naming to the point... if it is liver disease, whether acute or chronic, it simply says liver disease... this leaves our patient history incomplete.”*

The other issue raised by participants is the problem of physician–patient interaction. Communication will be hampered by an increase in provider screen stare, keyboarding, quietness, and closed body posture. A 29-year-old male participant expressed the following:

*“I believe that using EMR will ruin the physician-patient interaction. The physician's focus will be on the system rather than the formation of a patient-physician rapport. As a result, the physicians will miss critical information from the patient's interview.”*

### 3.7. Taking an EMR Training

The third point brought up by participants was the need of EMR training. Prior to system adoption, the majority of responders stressed the need of attending an EMR training. Furthermore, the majority of them thought that the EMR training they received had shifted their mindset about it. A 40-year-old male participant put it like way:

*“I took EMR training for two weeks and discovered that an EMR system would make medical work easier and reduce physicians' workload.”*

### 3.8. Computer Access at Work Place

From the interview with the respondents, the potential for health information exchange to promote health and minimize poor outcomes owing to manual documentation was unequivocally acknowledged as a justification for utilizing and supporting EMR system adoption by a broad range of participants. Participants who have access to a computer at their workplace believe that electronic health information sharing has a positive impact on their health. The following were the thoughts of a 36-year-old male participant:

*“At work, I have access to a computer. It's where I go to read about the problems I've had while providing care. This improves my trustworthiness with patients as well as my general efficiency in the workplace. As a result, by incorporating clinical decision support systems into EMRs, medical errors will be reduced, and advanced medical care and treatment will be improved.”*

The article "Physicians' Attitude towards Electronic Medical Record Systems: An Input for Future Implementers" was published in 2021. Journal: Biomed Res Int.

## 4. Discussion

This study examines physicians' attitudes about electronic medical record systems at referral hospitals in Ethiopia's Amhara regional state. We discovered major predictor variables for physicians' attitude towards electronic medical record systems, such as computer ownership, EMR training, computer literacy, lack of prior EMR experience, computer access at work, and physician involvement in EMR activities. Furthermore, the findings from in-depth interviews with key informants were found to be consistent with the quantitative findings.

This study revealed that more than 58 percent of the respondents scored above average on the provided fifteen Likert items. The finding is in line with the studies done in Ethiopia, North Gondar hospitals 54.6% [14], Aider referral hospital 56.1% [15], and Makkah region, Saudi Arabia 52.8% [33]. However, the result of this study demonstrated that physicians' positive attitude towards EMR was lower than studies done in Istanbul, Turkey 97% [36], India 80% [37], and Africa, Nigeria 67.2% [38]. The difference might be physicians who are working at high-resource countries and who have computer experience in their day-to-day life could understand the relative advantage of electronic medical record systems in health care.

The study also found factors influencing physicians' attitudes about electronic medical record systems. Physicians' computer literacy, ability to use Microsoft Office, and internet navigation were all favorable predictors of their attitude towards EMR systems. This finding is supported by studies conducted in California, America [39], Tamil Nadue, India [40], and Malaysia [41]. The possible reason for this could be that being computer literate had a direct influence on health professionals' views on computer-based system use.

The physicians' prior experience with the previously deployed EMR system and their attitude about the system were shown to be inversely related. This finding appeared to be consistent with studies done in Nairobi, Kenya [42] and found in the contrary with study done among Canadian physicians [43]. The reason might be the previously introduced EMR system had poor system design and used unstandardized medical terminologies.

Taking EMR system training was a good factor to changing the attitude about the EMR system. Physicians who received EMR training had a more positive attitude than physicians who did not get EMR training. And studies conducted in aider referral hospital and Addis Ababa suggested that taking training changes the attitude and motivation of physicians towards electronic medical record systems [9, 15]. This might be because physicians who got EMR training had more knowledge about the system than their colleagues, which improved their attitude and motivation towards the system.

The article "Physicians' Attitude towards Electronic Medical Record Systems: An Input for Future Implementers" was published in 2021. Journal: Biomed Res Int.

Computer access at workplace and having personal computer at home had also a statistical association with physician's attitude towards EMR. Physicians who have computer access at workplace and personal computer at home were found a positive predictive factor to have a positive attitude towards the EMR system. This result is consistent with other studies done in Harari region, Ethiopia [44], Tanzania [45], Korea [28], and Iran [46]. The probable reason for this might be physicians who have computer access could be more familiar towards computer-based information systems and could increase their belief towards EMR.

## 5. Conclusion

According to the findings of this study, physicians' attitudes regarding EMR were moderate in the studied region. There was a favorable relationship between computer ownership, computer literacy, lack of experience with maladapted EMR systems, EMR training, and computer access at work and attitude towards EMRs. Improving computer access at work, EMR training, and basic computer literacy are all necessary to enhance physicians' attitudes about EMR systems. One of the most important conclusions given in this study is that of poorly suited EMR systems. People who were exposed to inadequate EMR systems during their initial experience with electronic information systems acquire an unfavorable attitude about EMRs. As a result, prior to installation, implementers and high-level managers should verify the EMR system's applicability.

## Figures and Tables

**Table 1:** Sociodemographic characteristics of physicians in Amhara regional state at five major referral hospitals, Ethiopia 2018 (*n* = 403).

Variables	Category	Frequency	Percent
Sex of the respondents	Female	65	16.1
	Male	338	83.9
Age of respondents	<30 years	132	32.8
	31-36 years	146	36.2
	≥37 years	125	31
Educational states	General practitioners	227	56.3
	Residents	70	17.4
	Specialists	106	26.3
Physicians' placement	Community	191	47.4
	Academic	212	52.6
Computer ownership	Yes	226	56.1
	No	177	43.9
Role of physicians	Administrative	22	5.5
	Health professional	381	94.5
Work experience	≥6 years	172	42.7
	<6 years	231	57.3
Working part-time at private	Yes	285	70.7
	No	118	29.3

**Table 2:** Technology-related variables of physicians in Amhara regional state at five major referral hospitals, Ethiopia, 2018 (*n* = 403).

Variables	Category	Frequency	Percent
Computer literacy	Yes	117	29.0
	No	286	71.0
Having previous EMR experience	Yes	185	45.9
	No	218	54.1
Having IT-related experience	Yes	298	73.9
	No	105	26.1
Prefer EMR than paper based	Yes	245	60.8
	No	158	39.2
Reason for preferring EMR (*n* = 245)	EMR is more secured	228	93
	EMR is time saving	189	77.1
	Store more data	209	85.3
	Easy to access data	214	87.3
	Easy to write report	106	43.2
Reason for not preferring EMR (*n* = 158)	EMR is time consuming	131	92.9
	EMR is difficult to use	124	78.5
	Needs computer skills	108	68.3
	Is electric dependent	120	75.9
Taking training on EMR	Yes	245	60.8
	No	158	39.2

The article "Physicians' Attitude towards Electronic Medical Record Systems: An Input for Future Implementers" was published in 2021. Journal: Biomed Res Int.

**Table 3:** Organizational-related variables at five major referral hospitals in Amhara region, Ethiopia, 2018 (*n* = 403).

Variables	Category	Frequency	Percent (%)
Computer access in working area:	No	191	47.4
	Yes	212	52.6
Purpose of computer use (*n* = 210):	Reading	195	92.8
	EMR data recording	37	17.6
	Report preparation	108	51.4
	Video accessing	143	68.1
	Internet access	191	90.9
Responsible person for EMR:	No	226	56.1
	Yes	177	43.9
ICT center for computer maintenance:	No	120	29.8
	Yes	283	70.2
Hospital support for EMR:	No	145	36.0
	Yes	258	64.0
Involve physicians in EMR activities:	No	168	41.7
	Yes	235	58.3
Internet access at workplace:	No	100	24.8
	Yes	303	75.2
Raise EMR issues during meeting:	No	135	33.5
	Yes	268	66.5

**Table 4:** The relationship between the predictors and physicians' attitudes about EMR at five main referral hospitals in Amhara regional state, Ethiopia, in March 2018 (*n* = 403).

Variable	All (403)	95% of CI	*P* value
Sex			
Female	65	-0.353, 0.110	0.303
Male	338		
Age			
<30	132		
31-36	146	-0.422, -0.023	0.029^∗^
>37	125		
Physicians' placement			
Academic	212	-0.142, 0.286	0.507
Community	191		
Computer ownership			
Yes	226	0.037, 0.458	0.021^∗^
No	177		
Work experience			
≥6 years	172	-0.290, 0.371	0.809
<6 years	231		
Computer literacy			
Yes	286	0.264, 0.713	0.0001^∗∗^
No	117		
Previous EMR experience			
Yes	185	-0.517, -0.121	0.002^∗^
No	218		
IT experience			
Yes	298	-0.138, 0.299	0.469
No	105		
Taking EMR training			
Yes	245	0.159, 0.559	0.0001^∗∗^
No	158		
Computer access at work			
Yes	212	0.141, 0.533	0.001^∗∗^
No	191		
ICT center at work			
Yes	283	-0.153, 0.277	0.572
No	120		
Internet access			
Yes	303	-0.054, 0.407	0.132
No	100		

^∗∗^*P* < 0.001, ^∗^*P* ≥ 0.001.

## Data Availability

Data will be available upon request from the corresponding author.

## Abbreviations

CI: Confidence interval
MOH: Ministry of Health
EMR: Electronic medical record
HIT: Health information technology
ICT: Information communication technology
SPSS: Statistical Package for the Social Science
UOG: University of Gondar.
